# SAG expression associates with COPB2-related signaling and a poorer prognosis in breast cancer

**DOI:** 10.18632/aging.102663

**Published:** 2020-01-11

**Authors:** Aiyu Liu, Shizhen Zhang, Weihan Li, Biao Xu, Rui Lei, Shengmei Zhu

**Affiliations:** 1 Department of Anesthesiology, The First Affiliated Hospital, Zhejiang University School of Medicine, Hangzhou 310009, Zhejiang, China; 2 Institute of Translational Medicine, Zhejiang University, School of Medicine, Hangzhou 310029, Zhejiang, China; 3 Department of Acupuncture and Moxibustion, The Third Affiliated Hospital of Zhejiang Chinese Medical University, Hangzhou, 310005, Zhejiang, China; 4 Departmant of Galactophore Surgery, The Second Affiliated Hospital of Guangzhou University of traditional Chinese Medicine, Guangdong 510120, China; 5 Departmant of Plastic Surgery, The First Affiliated Hospital, Zhejiang University School of Medicine, Hangzhou 310009, ZhejiangChina

**Keywords:** SAG, COPB2, prognosis, proliferation, breast cancer

## Abstract

SAG is an essential RING component of the Cullin-RING ligase (CRL) E3 ubiquitin ligase complex, which regulates diverse signaling pathways and biological processes, including cell apoptosis, embryonic development, angiogenesis, and tumorigenesis. In the present study, we revealed that SAG gene expression is upregulated in breast cancer cells and that SAG overexpression is associated with significant poorer survival in breast cancer, especially the luminal A subtype. We also detected highly correlated co-overexpression of SAG and COPB2 in breast cancers. Subsequent *in vitro* experiments demonstrated that SAG and COPB2 act cooperatively to stimulate breast cancer cell proliferation, migration and invasion. Our findings suggest that levels of SAG and COPB2 expression may be useful prognostic indicators in breast cancers and that SAG may be involved in COPB2-related signaling during breast cancer development.

## INTRODUCTION

SAG (Sensitive to Apoptosis Gene), also known as RNF7 (RING finger protein-7) or ROC2 (Regulator of cullins-2), was originally identified as a redox inducible antioxidant protein [1], but was later characterized as one of the RBX/ROC RING component of CRL/E3 ubiquitin ligases [2]. Functioning as an antioxidant, SAG inhibits apoptosis induced by a variety of stimuli both *in vitro* and *in vivo* [1–5]*.* It is expressed ubiquitously in human tissues, especially tissues in which oxygen consumption is high, such as heart, skeletal muscle, and testis [6]. As a component of CRL/E3 ubiquitin ligase, on the other hand, SAG exhibits E3 ubiquitin ligase activity to promote the ubiquitylation and subsequent degradation of various cellular proteins, including p27, pro-caspase-3, HIF-1α, NOXA [7–10].

Because SAG/E3 targets several tumor suppressors for degradation, it is regarded as an oncoprotein [6]. Transgenic expression of *SAG* in mouse skin impairs tumor formation at early stages by targeting c-Jun/AP1 for degradation, whereas it promoted tumor growth at later stages by targeting IκBα to activate NF-κB [11]. Moreover, *SAG* knockout suppresses *Kras*^G12D^-driven lung tumorigenesis, suggesting *SAG* is a *Kras*-cooperating oncogene that promotes lung tumorigenesis [12]. Conversely, SAG is reportedly overexpressed in primary colon carcinomas and prostate cancers [13, 14], and an association between SAG overexpression and poor survival has been reported in lung cancers [12, 15]. It remains unclear, however, whether SAG expression is involved in breast tumorigenesis.

The coatomer protein complex subunit (COPB2), also known as Beta-Cop, P102 or Coatomer Protein Complex Subunit Beta Prime, is a subunit of the cytoplasmic protein complex that makes up the coat of non-clathrin-coated vesicles and is crucial for vesicular trafficking and Golgi budding [16]. Recently, the critical role of COPB2 in the tumorigenesis in several human cancers has attracted attention [17, 18]. For example, higher COPB2 expression is associated with lymph node metastasis of breast cancer, while COPB2 knockdown inhibits breast cancer cell proliferation and metastasis [19]. However, the related signaling pathways via which COPB2 is controlled during tumorigenesis are rarely investigated.

In the present study, we endeavored to pool public genomic data to assess the association between SAG expression and prognosis in breast cancer. Our findings show that SAG is associated with poorer survival in breast cancer, especially the luminal A subtype, and that there is highly correlated co-overexpression of SAG and COPB2 in breast cancers.

## RESULTS

### SAG expression is increased in breast cancers

Using bc-GenEx-Miner 4.3, we first analyzed the SAG expression profile across different breast cancer subtypes. As expected, SAG expression was significantly higher in breast cancer tissues than in normal breast-like tissues (Figure 1A). In addition, subgroup analysis revealed that SAG expression was associated with estrogen receptor (ER) and human epidermal growth factor 2 (HER2) expression status, but not with progesterone receptor (PR), triple-negative, or lymph node status (Figure 1B–1F). Because SAG is regarded as an oncoprotein and significantly associated with poor prognosis for several human cancers, we also used bc-GenExMiner to investigate whether SAG overexpression was associated with survival of breast cancer patients. The Kaplan-Meier curves showed that higher SAG expression correlated with poorer survival in breast cancer (Figure 1G). Moreover, another online public survival analysis tool (KM-plot) [20] confirmed that there was a trend in which elevated SAG expression was related to a poorer prognosis, though it did not reach statistical significance (Figure 1H).

**Figure 1:** **SAG is upregulated in breast cancer and associated with a poorer prognosis.** (**A**) Box plots showing SAG mRNA expression in the indicated breast cancer subtypes. (**B**–**F**) Box plots showing SAG mRNA expression in breast cancers characterized based on ER, PR, HER2, triple-negative, and nodal status. The Kaplan-Meier curves for SAG expression in breast cancer were constructed using UCSC bc-GenExMiner 4.3 (**G**) or KM-plot (**H**).

### Elevated SAG expression is associated with poor prognosis for lumina A breast cancers

To assess the relationship between SAG expression and prognosis in different breast cancer subtypes, Kaplan-Meier survival analyses were performed with four breast cancer subtypes using bc-GenExMiner 4.3. The results showed that high SAG expression was associated with poorer survival in patients with the luminal A subtype, but not the luminal B, HER2-overexpressing or basal-like subtype (Figure 2A–2C). These results were also confirmed using KM-plot, which indicated that SAG overexpression was associated with poorer survival only in lumina A type breast cancers (Figure 2D–2F).

**Figure 2:** **High expression of SAG mRNA correlated with poor outcomes in luminal A breast cancer.** Kaplan-Meier survival analysis performed using bc-GenExMiner 4.3 shows the relationship between SAG expression and survival in luminal A (**A**), luminal B (**B**), HER2-expressing (**C**) and basal-like (**D**) breast cancers. These data were re-analyzed and confirmed using KM-plot (**E**–**H**).

### SAG may be involved in COPB2-related signaling pathways

Given the apparent involvement of SAG in malignant behavior of breast cancer, we next investigated the signaling pathways in which SAG may be involved. Using the cBioPortal for Cancer Genomics with breast cancer data from The Cancer Genome Atlas (TCGA) database, 10 candidate genes were identified that positively correlated with SAG expression (Figure 3A). Among them, COBP2 is reportedly overexpressed in several human sarcomas and neoplastic tissues [21]. COPB2 also reportedly promotes lung cancer cell proliferation and tumorigenesis by upregulating YAP1 expression [18], and silencing COBP2 significantly inhibits cell proliferation and induces apoptosis in cholangiocellular carcinomas [22]. To further clarify the relationship between SAG and COPB2, we used the CBioPortal to examine the RNAseq data in a breast cancer cohort and showed that SAG is co-upregulated with COPB2 (Figure 3B.). The heat map generated using the UCSC Xena browser confirmed that SAG is highly co-upregulated with COPB2 in breast cancers (Figure 3C). Moreover, this relationship between SAG and COPB2 was most significant in luminal B breast cancers (Figure 3D–3G).

**Figure 3:** **SAG may be involved in COPB2-related signaling.** (**A**) Top 10 genes positively correlated to SAG expression in breast cancer. (**B**) Correlation between SAG and COPB2 analyzed using cBioPortal for Cancer Genomics. (**C**) Heat map of the correlation between SAG and COPB2. Co-expression of SAG and COPB2 in luminal A (**D**), luminal B (**E**), HER2-expressing (**F**) and basal-like (**G**) breast cancers analyzed using bc-GenExMiner 4.3.

### COPB2 and SAG are both upregulated in breast cancer cells

To confirm whether there is a positive correlation between SAG and COPB2 expression. We used the Human Protein Atlas (https://www.proteinatlas.org) to assess the relative levels of SAG and COPB2 expression in a large number of cell lines from different types of human cancers. The results showed that the level of SAG expression correlated positively with the level of COPB2 expression in several human cancer cell lines (Figure 4A, 4B). We then used RT-qPCR to measure the relative levels of SAG and COPB2 expression in three breast cancer cell lines (MCF-7, SKBR-3 and T47d) and in a normal breast cell line (MCF-10A). We found that gene expression of both SAG and COPB2 was higher in all three breast cancer cell lines than in normal breast tissue cells (Figure 4C, 4D). In SKBR-3 and T47d cells, we were able to knock down expression of both SAG and COPB2 using targeted siRNAs (Figure 4E and 4F).

**Figure 4:** **Levels of SAG and COPB2 expression in breast cancer cell lines.** (**A**) SAG expression in human cancer cells from a cohort in TCGA database. (**B**) COPB2 expression in human cancer cells from a cohort in TCGA database. (**C**–**D**) RT-qPCR analysis of the relative levels of SAG expression in SKBR3 (**C**) and T47D (**D**) cells. Levels of SAG and COPB2 mRNA were significantly decreased following transfection with the indicated siRNAs in SKBR3 (**E**) and T47D (**F**) cells. (*P < 0.05).

### SAG and COPB2 act cooperatively to enhance breast cancer cell proliferation

Because both SAG and COPB2 exert pro-proliferative effects in several human cancers [10, 12, 19, 23], we wanted to determinate how SAG and COPB2 knockdown influenced breast cancer cell proliferation, and whether SAG and COPB2 acted cooperatively to affect cell proliferation. As expected, knocking down SAG or COPB2 inhibited breast cancer cell proliferation (Figure 5). Conversely, ectopic overexpression of SAG in SKBR-3 or T47d breast cancer cells enhanced the cells’ proliferative potential. Notably, COPB2 knockdown in SAG- overexpressing cells completely reversed the enhanced cell growth induced by SAG overexpression. These results suggest that COPB2-related signaling is involved in SAG’s pro-proliferative effect.

**Figure 5:** **SAG and COPB2 knockdown inhibits breast cancer cell proliferation.** (**A**, **B**) CCK-8 assays measuring breast cancer cell proliferation following SAG or COPB2 knockdown. (**C**, **D**) CCK-8 assays measuring breast cancer cell proliferation following transfection of Flag-SAG with and without siRNA targeting COPB2. (*P < 0.05).

### SAG-COBP2 regulates breast cancer cell migration and invasion

To further evaluate the oncogenic effects of SAG and COPB2 in breast cancer cells, we performed a set of transwell migration and invasion assays. We found that SAG or COPB2 knockdown significantly inhibited breast cancer cell migration and invasion as compared to the control group (Figure 6A–6C), while ectopic overexpression of SAG slightly enhanced breast cancer cell migration and invasion. Most importantly, COPB2 knockdown in SAG-overexpressing cells suppressed the enhanced migration and invasion induced by SAG (Figure 6A–6C).

**Figure 6:** **Downregulation of SAG or COPB2 inhibited breast cancer cell migration and invasion.** (**A**) Representative images of migrated cells following transfection with the indicated genes. (**B**) Columns representing the relative number of migrated cells in the different groups. (**C**) Columns representing the relative number of invading cells in the different groups. (*P < 0.05).

## DISCUSSION

SAG reportedly functions as a redox-inducible antioxidant protein and as a RING component of CRL controlling the turnover of numerous substrates involved in cell proliferation, apoptosis, and tumorigenesis [1, 2]. In lung cancer, it is known that SAG acts as an onco-cooperating gene required for tumorigenesis induced by a mutant Kras [12], that it is significantly overexpressed in lung cancer tissues, and that its expression correlates with poor patient prognosis [15]. Knocking down SAG inhibits lung cancer cell proliferation, *in vitro* and in *vivo*, and contributes to the recovery of radiation sensitivity in radiation-resistant cancer cells [10]. By contrast, to our knowledge there have been no studies examining SAG’s actions in breast cancer. In the present study, however, we showed that levels of SAG mRNA are significantly higher in breast cancer tissues than in normal breast-like tissues and that increased SAG expression is associated with the ER and HER2 expression status of breast cancer. In addition, we provide evidence that SAG exerts a pro-proliferative effect in breast cancer cells and that its overexpression is associated with unfavorable prognosis in breast cancer.

We also observed that COPB2 is highly upregulated along with SAG in breast cancers. COPB2 is a subunit of the Golgi coatomer complex, which acts as a mediator for transport of proteins from the endoplasmic reticulum to the Golgi apparatus during protein biosynthesis [16]. COPB2 expression levels are upregulated in several human cancers and are associated with their prognosis [19, 23, 24]. Furthermore, COPB2 knockdown leads to inhibition of cell proliferation, cell cycle arrest, and induction of apoptosis [19, 23, 24]. Notably, one recent qRT-PCR analysis revealed that COPB2 mRNA levels were significantly higher in breast cancer tissues than in normal tissues, suggesting COPB2 is a potential tumor oncogene in breast cancer [19]. Here, we confirmed upregulation of COPB2 in three breast cancer cell lines, but not in normal breast epithelial cells. In lung cancer cells, COPB2 inhibits apoptosis and promotes cell proliferation and tumorigenesis through up-regulation of YAP1 expression [18], while COPB2 knockdown in gastric cancer cells suppresses cell proliferation and promotes apoptosis by repressing the RTK signaling cascade [23]. In the present study, we found that COPB2 is upregulated along with SAG in breast cancers and that both are highly expressed in breast cancer cell lines. Moreover, COPB2 knockdown abolished SAG-induced breast cancer cell proliferation and invasion, which strongly suggests COPB2 signaling is involved in the mechanism underlying the oncogenic effect of SAG.

Taken together, our findings indicate that expression of SAG and COPB2 may be a useful prognostic indicator in breast cancer. Moreover, SAG may be involved in a COPB2-related signaling pathway that plays an oncogenic role in breast cancer.

## MATERIALS AND METHODS

### Bioinformatic analysis of gene expression in breast cancer

The mRNA expression of genes in various breast cancer subtypes was assessed using an online platform for gene expressive and prognostic analyses (Breast Cancer Gene-Expression Miner Version 5.0), which includes published annotated genomic data from 5609 breast cancer patients [25, 26]. The mRNA expression of genes in various human cancer cell lines was analyzed using the Human Protein Atlas (https://www.proteinatlas.org).

### Survival analysis based on public data

The relationship between *SAG* or *COPB2* expression and survival in different breast cancer subtypes was analyzed using bc-GenExMiner 4.3 [25]. The survival relationships obtained were verified by re-analysis using the online Kaplan-Meier plotter database, which was established using gene microarray data and survival information downloaded from the Gene Expression Omnibus (GEO) [27].

### Bioinformatic analysis of SAG-related genes in breast cancer

The top 10 SAG-related genes co-upregulated with SAG were identified using the cBioPortal for Cancer Genomics. In addition, the UCSC Xena browser (http://xena.ucsc.edu/) was used to produce expression heat maps for SAG and COPB2.

### Cell culture

The MCF-10A normal breast cell line and MCF-1, SK-BR-3, and T-47D breast cancer cell lines were purchased from Shanghai Cell Biology, Institute of the Chinese Academy of Sciences (Shanghai, People's Republic of China). MCF-1 and SK-BR-3 cells were cultured in Dulbecco's modified Eagle's medium (DMEM; Gibco, Grand Island, NY, USA) supplemented with 10% fetal bovine serum (FBS; Gibco, Grand Island, NY, USA) and 100 IU/ml penicillin, and 100 μg/ml streptomycin. T-47D cells were cultured in Roswell Park Memorial Institute-1640 medium (Gibco, Grand Island, NY, USA) with 10% FBS (Gibco). MCF-10A cells were cultured in DMEM-F12 (Gibco) supplemented with 100 μg/mL streptomycin, 100 U/mL penicillin, 20 ng/mL epidermal growth factor (EGF), 2 mmol/L L-glutamine and 10% FBS (Gibco). All cell lines were maintained in a standard cell culture incubator (Thermo, Waltham, MA, USA) at 37°C with 5% CO_2_.

### RNA inference and plasmid overexpression

siRNAs targeting COPB2 and SAG were purchased from Shanghai Gene Pharma (Shanghai, China). The sequences were as follows: for COPB2, CCCAUUAUGUUAUGCAGAUTT; for SAG, CCTGTGGGTGAAACAGAACAA. Following the manufacturer's instructions, the siRNA was transfected into cells using GeneMute transfection reagent. After 48 h, the transfected cells were harvested for subsequent RNA expression analysis. Flag-SAG plasmid was transfected as described previously [28].

### CCK-8 assays

Cells were transfected with the indicated target siRNAs or plasmids for 24 h, after which they were seeded into 96-well plates to a density of about 1500 cells/well. After 24, 48, 72 and 96 h, cell viability was assessed based on the absorbance of 450 nm using a CCK-8 assay kit.

### Cell invasion and migration assays

The cells’ capacity for migration and invasion were assessed using transwell chambers according to the manufacturer's instructions (Corning Costar Corp., Cambridge, USA). Briefly, after transfecting cells with indicated siRNAs or plasmids for 48 h, about 3×10^4^ cells/well of cells were transferred into the upper chambers, while the lower chambers were filled with 600 ml of medium containing with 20% FBS. After 24 h, the filters separating the upper and lower chambers were carefully removed, and the cells were fixed with 4% paraformaldehyde and stained with Giemsa and eosin. Cells that had migrated to the underside of the filters were counted under a light microscope.

### Statistical analysis

Statistical analyses were done using the SPSS version 23.0 (SPSS, Inc, Chicago, IL) and GraphPad Prism version 6.0 (GraphPad Software, Inc, La Jolla, CA) statistical software packages. Comparisons between groups were made using Student's t-test (two-tailed) or one-way analysis of variance with Dunnett’s method for multiple comparisons. Values of *P*<0.05 was considered statistically significant.
